# Sentiment Analysis Based on the Nursing Notes on In-Hospital 28-Day Mortality of Sepsis Patients Utilizing the MIMIC-III Database

**DOI:** 10.1155/2021/3440778

**Published:** 2021-10-13

**Authors:** Qiaoyan Gao, Dandan Wang, Pingping Sun, Xiaorong Luan, Wenfeng Wang

**Affiliations:** ^1^Nursing Department, Weihai Central Hospital, Weihai, 264400 Shandong, China; ^2^Nursing Department, Qilu Hospital of Shandong University, Jinan, 250012 Shandong, China; ^3^School of Science, Shanghai Institute of Technology, Shanghai 201418, China; ^4^International Academy of Visual Art and Engineering, London E16 1AH, UK; ^5^Interscience Institute of Management and Technology, Bhubaneswar 752054, India

## Abstract

In medical visualization, nursing notes contain rich information about a patient's pathological condition. However, they are not widely used in the prediction of clinical outcomes. With advances in the processing of natural language, information begins to be extracted from large-scale unstructured data like nursing notes. This study extracted sentiment information in nursing notes and explored its association with in-hospital 28-day mortality in sepsis patients. The data of patients and nursing notes were extracted from the MIMIC-III database. A COX proportional hazard model was used to analyze the relationship between sentiment scores in nursing notes and in-hospital 28-day mortality. Based on the COX model, the individual prognostic index (PI) was calculated, and then, survival was analyzed. Among eligible 1851 sepsis patients, 580 cases suffered from in-hospital 28-day mortality (dead group), while 1271 survived (survived group). Significant differences were shown between two groups in sentiment polarity, Simplified Acute Physiology Score II (SAPS-II) score, age, and intensive care unit (ICU) type (all *P* < 0.001). Multivariate COX analysis exhibited that sentiment polarity (HR: 0.499, 95% CI: 0.409-0.610, *P* < 0.001) and sentiment subjectivity (HR: 0.710, 95% CI: 0.559-0.902, *P* = 0.005) were inversely associated with in-hospital 28-day mortality, while the SAPS-II score (HR: 1.034, 95% CI: 1.029-1.040, *P* < 0.001) was positively correlated with in-hospital 28-day mortality. The median death time of patients with PI ≥ 0.561 was significantly earlier than that of patients with PI < 0.561 (13.5 *vs*. 49.8 days, *P* < 0.001). In conclusion, sentiments in nursing notes are associated with the in-hospital 28-day mortality and survival of sepsis patients.

## 1. Introduction

Sepsis, a syndrome of life-threatening physiologic, pathologic, and biochemical dysfunction due to uncontrolled responses to infection, is one of the leading causes of deaths in intensive care units (ICUs) [1]. Despite advances in care, sepsis remains among the costliest diseases, approximately accounting for over 20 billion (5.2%) of total United States (US) hospital costs [2]. In the US, admission for sepsis has overtaken that for stroke and myocardial infarction [3]. According to statistics, the prevalence of sepsis is up to 535 cases per 100 100,000 person-years and on the rise [4]. Population-level epidemiological data show that there are 31.5 million cases of sepsis and 19.4 million cases of severe sepsis worldwide, with 5.3 million potential deaths each year [5], and the in-hospital mortality reaches up to 25%-30% [6].

Currently, severity of illness scores (SOI) is usually used to predict mortality in ICUs. The SOI system is established according to the coded data of patients' demographics, vital signs, and laboratory results usually accessed from the electronic health records, but there also exist unstructured data in the electronic health records, such as clinical notes written by clinicians which are not frequently used for predicting mortality [7]. Studies have demonstrated that clinicians can properly predict mortality in ICUs [8, 9]. Thus, their notes may provide some important information for patients' health status assessment. A previous study showed that the sentiment of clinicians towards patients could be evaluated by sentiment analysis, a method to classify the subjective properties of written text [10]. Sentiments measured in clinical notes are different according to demographic features and clinical outcomes [10]. There are studies suggesting that sentiments measured in clinical notes are associated with hospital readmission and mortality [11, 12].

In this study, we investigated the association of sentiments in nursing notes with the in-hospital 28-day mortality of sepsis patients based on the Medical Information Mart for Intensive Care (MIMIC-III) database, a freely accessible critical care database, aimed at providing some evidence for the improvement of patients' outcomes in ICUs.

## 2. Methods

### 2.1. Study Population

The data of patients and nursing notes were accessed from the MIMIC-III database developed by the MIT Lab for computational physiology. As an openly available dataset, MIMIC-III contains deidentified health data related to approximately 60,000 ICU admissions, including demographics, laboratory tests, medications, vital signs, transcribed nursing notes, diagnostic and procedure codes, fluid balance, length of stay, survival data, and others [13]. The inclusion criteria of this study were as follows: (1) patients diagnosed with sepsis, severe sepsis, and septic shock (International Classification of Diseases 9 (ICD-9) codes: 99591, 99592, and 78552) in the MIMIC-III database and (2) 15 years old or above at hospital admission. The exclusion criteria were as follows: (1) notes identified by physicians as errors, (2) notes written less than 12 hours before the time of death, and (3) patients without any data of nursing notes.

The data used in this study were obtained from the MIMIC-III database (https://mimic.physionet.org/), an openly available dataset. The data collection in the MIMIC-III was approved by the Ethics Review Board of the Beth Israel Deaconess Medical Center, and all private information has been desensitized.

### 2.2. Sentiment Analysis

Two techniques (syntactic and sematic) are mainly used to classify and compute the sentiment polarity in text [14]. A semantic approach means that the sentiment is extracted based on text meaning and is commonly obtained using a classifier [14]. To make inferences based on text structural features, this study employed a syntactic technique to extract sentiments.

Both the Python programming language and TextBlob natural language processing library were adopted to compute sentiment scores for the nursing notes [15]. The sentiment of text strings was computed using the pattern module in TextBlob. The pattern comprised a lexicon for various English language adverbs and adjectives able to be mapped to three dimensions of sentiment scores: polarity, subjectivity, and intensity [16]. The sentiment polarity was returned using TextBlob with a score from -1 to 1, and the sentiment subjectivity was returned with a score from 0 to 1. Higher scores showed more positive, subjective sentiments. In this study, both the polarity score and subjectivity score were assigned for each nursing note, and the scores were computed through establishment of a TextBlob object initialized with nursing note strings and extraction of sentiment attributes from the object [7]. The mean scores of sentiment polarity and subjectivity in nursing notes written during hospitalization were calculated for the first hospital admission of each patient and then used as predictors in the model of this study. For an example of sentiment polarity scores using TextBlob, see Table 1.

### 2.3. Mortality and Survival Assessment

As a common predictor of ICU mortality, Simplified Acute Physiology Score II (SAPS-II) is a composite score, including 17 variables (age, 12 physiology variables, type of admission, and 3 underlying disease variables) [17]. In this study, the SAPS-II score was calculated by the data from the MIMIC-III database and SQL scripts in the MIT Lab for computational physiology git repository. Additionally, gender and ICU type were also enrolled as variables because they were freely accessed from the MIMIC-III database, but not involved in SAPS-II. Survival was defined as the number of days from hospital admission to death or right-censoring time.

### 2.4. Statistical Analysis

Statistical analysis was performed using SPSS 22.0 software (IBM Corp., Armonk, NY, USA) and Python text analysis (version 3.7). Normally distributed data were compared by the *t*-test and manifested as mean ± standard deviation ($\overset{¯}{x}\pm s$); abnormally distributed data were compared with the Mann-Whitney *U* rank-sum test and presented as median and quartile (*M* (Q1, Q3)). Enumeration data were compared by the *χ*^2^ test, with *n* (%) as the manifestation. The COX proportional hazard model was used to analyze the relationship between sentiment scores in nursing notes and the in-hospital 28-day mortality of sepsis patients. The size power of our study was 0.858.

The common type of the COX model was *h*(*t*) = *h*0(*t*)exp(*X*′*β*), in which *h*0(*t*) and *h*(*t*) represented the datum risk function and the risk function at *t* time point, respectively, *X* was the covariate vector quantity, and *β* was the unknown vector quantity of the regression coefficient. The formula of the individual prognostic index (PI) was PI = *X*1*β*1 + *X*2*β*2 + ⋯+*Xkβk*. Based on the COX model, the individual PI was calculated. The greater the individual PI, the worse the prognosis. The survival curves were compared using a log-rank test. Box plot, histogram, and forest plot in our study were plotted with Python software. The power analysis was carried out to assess the statistical power (1 − *β*) using PASS 15.0 software (NCSS, LLC). The results showed that the power values of the sentiment polarity score and sentiment subjectivity score were all 1.000. It was indicated that our findings performed well reliability. A significant difference was shown at *P* < 0.05.

## 3. Results

### 3.1. Baseline Characteristics of the Study Population

In the MIMIC-III database, there were a total of 3567 patients admitted to the ICU. Of these patients, 1128 patients without sepsis, 356 cases lacking sentiment polarity and subjectivity scores, 172 with missing SAPS-II, and 60 with missing survival data were excluded. Totally, 1851 sepsis patients were eligible for the study, among whom 580 patients suffered from in-hospital 28-day mortality from the date of ICU admission (dead group), while 1271 patients survived (survived group). The baseline characteristics of the two groups were compared as shown in Table 2, and the flowchart is presented in Figure 1.

The sentiment polarity score of patients in the survived group was significantly higher than that in the dead group (*P* < 0.001), while the SAPS-II score was notably lower than that in the dead group (*P* < 0.001) (Table 2, Figure 2). The differences were significant between the two groups in age (*P* < 0.001) and ICU type (*P* < 0.001), but not in the sentiment subjectivity score (*P* = 0.340) and gender (*P* = 0.757) (Table 2, Figure 3).

### 3.2. COX Regression Analysis of the Association between Sentiments and 28-Day Mortality

As shown in Table 3, univariate analysis showed an inverse association between sentiment polarity and 28-day mortality (hazard ratio (HR): 0.458, 95% confidence interval (95% CI): 0.401-0.524, *P* < 0.001) and no association between sentiment subjectivity and 28-day mortality (HR: 0.863, 95% CI: 0.657-1.133, *P* = 0.289). The risk of 28-day mortality in sepsis patients would increase 0.04 times when 1 point in the SAPS-II score was increased each time (HR: 1.040, 95% CI: 1.036-1.045, *P* < 0.001). There was no association between gender and 28-day mortality (HR: 1.104, 95% CI: 0.936-1.301, *P* = 0.240).

In multivariate analysis, it was observed that both sentiment polarity (HR: 0.499, 95% CI: 0.409-0.610, *P* < 0.001) and sentiment subjectivity (HR: 0.710, 95% CI: 0.559-0.902, *P* = 0.005) were inversely associated with in-hospital 28-day mortality, while the SAPS-II score (HR: 1.034, 95% CI: 1.029-1.040, *P* < 0.001) was positively correlated with in-hospital 28-day mortality. The patients aged ≥80 years had an increased risk of in-hospital 28-day mortality compared with those aged <40 years (HR: 1.612, 95% CI: 1.032-2.520, *P* = 0.036). There were no differences in in-hospital 28-day mortality between the age of 40-59 (HR: 1.217, 95% CI: 0.781-1.886, *P* = 0.385), 60-69 (HR: 1.479, 95% CI: 0.943-2.321, *P* = 0.089), 70-74 (HR: 1.048, 95% CI: 0.637-1.723, *P* = 0.854), 75-79 (HR: 1.030, 95% CI: 0.629-1.687, *P* = 0.906), and <40 years. In addition, no significant difference was found between gender and 28-day mortality (HR: 1.104, 95% CI: 0.934-1.306, *P* = 0.245). Patients that stayed in the trauma/surgical intensive care unit (TSICU) were least likely to die within 28 days after admission (HR: 0.280, 95% CI: 0.190-0.414, *P* < 0.001) (Table 3, Figure 4).

### 3.3. Survival Analysis

According to the individual PI, patients were assigned into the high-risk group (PI ≥ 0.561) and the low- and middle-risk group (PI < 0.561), and the survival curves are illustrated in Figure 5. It could be observed that the median death time of the high-risk group was significantly earlier than that of the low- and middle-risk group (13.5 *vs*. 49.8 days, *P* < 0.001).

## 4. Discussion

In the present study, a total of 1851 sepsis patients were eligible according to inclusion and exclusion criteria, among whom 580 cases suffered from in-hospital 28-day mortality, while 1271 cases survived. Multivariate COX analysis showed that sentiment polarity and sentiment subjectivity were inversely associated with in-hospital 28-day mortality. Based on the quartiles of the individual PI, patients were assigned into the high-risk group and the low- and middle-risk group. Survival analysis indicated that the high-risk group had earlier median death time compared with the low- and middle-risk group. These all suggested that the quantitative measurement of sentiments in nursing notes was associated with the in-hospital 28-day mortality and survival of sepsis patients; nursing notes containing rich information may serve as a potential predictor of clinical outcomes in the ICU.

To the best of our knowledge, brief fragments of the text are conducive to reflecting the author's feelings about a given topic. Recently, language processing tools have been developed and allow the characterization of feelings, such as the sentiment in text documents [18]. Sentiment is usually described as the relative positivity or polarity of a text string and is measured by a number from -1 (very negative) to 1 (very positive) [14]. It can also be interpreted as the estimated probability of “positive” or “negative” through a classifier. Sentiment analysis permits us to gain insights into the clinicians' emotions and attitudes towards patients through the subjective expressions made by clinicians in the text of clinical notes, thus contributing to the prediction of patients' outcomes [19–22]. In health-related fields, sentiment analysis has been widely applied to Cancer Survivors Network (CSN) breast and colorectal cancer discussion posts [23], health reforms on Twitter [24], encounter notes of patients with critical illness [25], etc. This study was aimed at identifying the association between sentiments in nursing notes and the in-hospital 28-day mortality of sepsis patients. The results exhibited that both sentiment polarity and sentiment subjectivity were inversely associated with in-hospital 28-day mortality, supported by the results of McCoy et al. that the sentiment measured in hospital discharge notes was related to hospital readmissions and mortality risk [11]. Based on the COX model, the patients with PI ≥ 0.561 were found to have a higher risk of death than those with PI < 0.561, highlighting the potential value of sentiments in survival analysis. A previous study has shown a strong association between sentiments and the risk of death even after adjustment for severity of illness and baseline information [25].

The superiority of the present study was that it was the first study to investigate the association between sentiments in nursing notes and the in-hospital 28-day mortality of sepsis patients. The nursing notes written less than 12 hours before the time of death were excluded, which made the results more reliable. However, the present study also had several limitations that should be cautiously interpreted. First, nursing notes from the MIMIC-III database with single-center samples may manifest different characteristics because of variations in clinicians, experience, training, or working environment, easily causing the results to be nongeneralizable. Second, the approach used to measure the sentiment in the present study was not the only approach available. Other techniques could produce different results, such as those based on the machine learning model to make semantic inferences. Third, the mean sentiment scores could only characterize the variations at the level of patients, but not at the levels of sentences, paragraphs, or documents. Forth, the nursing notes were recorded by caregivers who are research nurses, medical doctors, or so on (available at https://mimic.mit.edu/docs/iii/tab les/caregivers/). It cannot be determined whether the sentiments based on nursing notes are based on past or personal experiences. Moreover, the subtle difference in sentiments was not obtained over time. In the future, the temporal mode of nursing notes will be examined to gain more insights.

## 5. Conclusions

Sentiments in nursing notes are associated with the in-hospital 28-day mortality and survival of sepsis patients, suggesting the importance of sentiments in nursing notes for the prediction of clinical outcomes in the ICU. Although predicting clinical outcomes is still a complex problem, the information extracted from unstructured data like nursing notes may contribute to further improving prediction performance.

## Figures and Tables

**Figure 1:** Flow diagram of patient screening from the MIMIC-III database.

**Figure 2:** Box plot of the score of sentiment polarity, sentiment subjectivity, and SAPS-II between two groups.

**Figure 3:** Histogram of the age, gender, and ICU type between survived and dead groups.

**Figure 4:** Forest plot of multivariate analysis of the association between sentiments and 28-day mortality.

**Figure 5:** Survival curve comparison of two groups according to the individual prognostic index.

**Table 1:** An example of sentiment polarity scores using TextBlob.

Excerpt text with deidentified patient information	Polarity score	Subjectivity score
New pt from ED,reffered from [∗∗Hospital3 1589∗∗],kc/o ESRD with HD, chronic diarrhea,c-diff,MRSA,presented with low BP treated with antibiotics,levophed,and dopamine,and transffered to [∗∗Hospital1 54∗∗] ED for further management,received 3lit FB IN ED,off dopa,on levophed and transffered to [∗∗Hospital Unit Name 44∗∗] for further management.VSS. ON NRBM sats 99%.having multiple sores on both legs and arms,amputated most of the fingers and toes. Pt not following with commands,not talking. Unable to assess orientation.	0.017	0.357

STATUS D: INTUBATED ON PROPOFOL GTT FOR COMFORT..FOLLOWS COMMANDS MOVES ALL EXTREM'S..K+'S DOWN A: PROPOFOL WEANED OFF & PT EXTUBATED WITHOUT PROB..ORAL NG DC'D.. SAT'S GOOD ON OFM @ 40%..STRONG COUGH..OOB TO CHAIR WITH 2 ASSISTS TOL WELL..A-LINE DC'D..K+ REPLETED..GOOD HUO..ABD SOFT WITH + BS'S R: STABLE P: [∗∗Month (only) 83∗∗] BE TRANSFERED TO FLOOR IF NEED BED PER DR [∗∗First Name (STitle) 349∗∗]..MONITOR K+'S & REPLETE AS NEEDED..LABS PER HO..CONTINUE WITH GOOD PULMONARY TOILET START CL LIQ'S AS TOL	0.101	0.522

See careview data and transfer note. Neuro: A&O x3. CV: Afib with controlled ventricular response, sbp 100-130's/50's. Pulm: RA sats 94-97%, lungs clear, pt occ productive of thick blood tinged sputum. GU: Uo 25-120cc hr/clr yellow, foley catheter dc'd at noon. GI: Taking house diet without difficulty. P: Chest CT today/?mass, pt to transfer to medical floor with goal to discharge home.	-0.050	0.215

**Table 2:** Baseline characteristics of survived and dead groups (*n* (%)).

Variables	Survived group (*n* = 1271)	Dead group (*n* = 580)	Total	*t*/*χ*^2^	*P*
Sentiment polarity score ($\overset{¯}{x}\pm s$)	0.051 ± 0.038	0.026 ± 0.040	0.043 ± 0.040	12.47	<0.001
Sentiment subjectivity score ($\overset{¯}{x}\pm s$)	0.377 ± 0.036	0.376 ± 0.040	0.377 ± 0.037	0.95	0.340
SAPS-II score ($\overset{¯}{x}\pm s$)	43.63 ± 15.51	57.27 ± 15.77	47.906 ± 16.825	17.44	<0.001
Age (years)				24.45	<0.001
<40	92 (7.20)	23 (4.00)	115 (6.20)		
40-59	330 (26.00)	143 (24.70)	473 (25.60)		
60-69	222 (17.50)	126 (21.70)	348 (18.80)		
70-74	152 (12.00)	53 (9.10)	205 (11.10)		
75-79	172 (13.50)	57 (9.80)	229 (12.40)		
≥80	303 (23.80)	178 (30.70)	481 (26.00)		
Gender				0.096	0.757
Female	573 (45.10)	257 (44.30)	830 (44.80)		
Male	698 (54.90)	323 (31.60)	1021 (55.20)		
ICU type				25.36	<0.001
CCU	51 (4.00)	48 (8.30)	99 (5.30)		
CSRU	36 (2.80)	25 (4.30)	61 (3.30)		
MICU	738 (58.10)	352 (60.70)	1 090 (58.90)		
SICU	284 (22.30)	96 (16.60)	380 (20.50)		
TSICU	162 (12.70)	59 (10.20)	221 (11.90)		

SAPS-II: Simplified Acute Physiology Score II; ICU: intensive care unit; CCU: coronary care unit; CSRU: cardiac surgery recovery unit; MICU: medical intensive care unit; SICU surgical intensive care unit; TSICU: trauma/surgical intensive care unit.

**Table 3:** COX regression analysis of the association between sentiments and 28-day mortality.

Variables	Univariate analysis		Multivariate analysis		
	HR (95% CI)	*P*	HR (95% CI)	*P*	*β*
Sentiment polarity score	0.458 (0.401, 0.524)	<0.001	0.499 (0.409, 0.610)	<0.001	-0.694
Sentiment subjectivity score	0.863 (0.657, 1.133)	0.289	0.710 (0.559, 0.902)	0.005	-0.342
SAPS-II score	1.040 (1.036, 1.045)	<0.001	1.034 (1.029, 1.040)	<0.001	0.034
Age (<40) (years)					
40-59	3.027 (1.955, 4.687)	<0.001	1.217 (0.781, 1.886)	0.385	0.196
60-69	1.462 (0.941, 2.272)	0.091	1.479 (0.943, 2.321)	0.089	0.391
70-74	2.074 (1.328, 3.238)	0.001	1.048 (0.637, 1.723)	0.854	0.047
75-79	1.584 (0.969, 2.591)	0.067	1.030 (0.629, 1.687)	0.906	0.030
≥80	1.721 (1.058, 2.799)	0.029	1.612 (1.032, 2.520)	0.036	0.478
Gender (female)					
Male	1.104 (0.936, 1.301)	0.240	1.104 (0.934, 1.306)	0.245	0.099
ICU type (CCU)					
CSRU	0.335 (0.206, 0.545)	<0.001	0.397 (0.243, 0.650)	<0.001	-0.923
MICU	0.475 (0.351, 0.643)	<0.001	0.527 (0.388, 0.715)	<0.001	-0.641
SICU	0.254 (0.179, 0.361)	<0.001	0.299 (0.210, 0.426)	<0.001	-1.208
TSICU	0.240 (0.163, 0.354)	<0.001	0.280 (0.190, 0.414)	<0.001	-1.272

SAPS-II: Simplified Acute Physiology Score II; ICU: intensive care unit; CCU: coronary care unit; CSRU: cardiac surgery recovery unit; MICU: medical intensive care unit; SICU: surgical intensive care unit; TSICU: trauma/surgical intensive care unit; HR: hazard ratio; 95% CI: 95% confidence interval.

## Data Availability

The data utilized to support the findings are available from the corresponding authors upon request. The data applied in the present study were from the MIMIC-III database (https://mimic.physionet.org/), a freely accessible database.

## Abbreviations

PI: Prognostic index
SAPS-II: Simplified Acute Physiology Score II
ICU: Intensive care unit
SOI: Severity of illness scores
MIMIC-III: Medical Information Mart for Intensive Care II
ICD-9: International Classification of Diseases 9
HR: Hazard ratio
TSICU: Trauma/surgical intensive care unit
CSN: Cancer Survivors Network.
